# A Retrospective Study of Lip Hemangiomas: Curative Effect of Oral Propranolol Combined with Topical Sclerotherapy

**DOI:** 10.1155/2022/6010458

**Published:** 2022-07-25

**Authors:** Jiaqi Ling, Kun Yang, Ran Huo, Dongsheng Zhang

**Affiliations:** ^1^Department of Plastic Surgery, Shandong Provincial Hospital, Cheeloo College of Medicine, Shandong University, Jinan, 250000 Shandong, China; ^2^Department of Plastic Surgery, Shandong Provincial Hospital Affiliated to Shandong First Medical University, Jinan, 250000 Shandong, China; ^3^Medical Science and Technology Innovation Center, Shandong First Medical University & Shandong Academy of Medical Sciences, China; ^4^Department of Stomatology, Shandong Provincial Hospital, Cheeloo College of Medicine, Shandong University, Jinan, 250000 Shandong, China; ^5^Department of Stomatology, Shandong Provincial Hospital Affiliated to Shandong First Medical University, Jinan, 250000 Shandong, China

## Abstract

**Objective:**

To analyze the therapeutic effect of oral propranolol combined with sclerotherapy of lauromacrogol and triamcinolone acetonide in the treatment of lip infantile hemangiomas (IHs).

**Methods:**

We recorded the demographic characteristics and lesions of 56 patients with lip IHs. The efficacy was evaluated by Achauer grade and VAS score in this study. Nonparametric test and Spearman correlation analysis were used to identify factors that might affect the curative effect of patients, and multivariate logistic regression analysis was used to further analyze the factors that affect the prognosis of patients with lip IH.

**Results:**

All 56 patients improved without serious complications after treatment. Univariate analysis showed that the age of the patients at the time of treatment initiation, the layer, classification, and volume of IH may influence the course and outcome of treatment. The logistic regression analysis further showed that the frequency of topical sclerotherapy was affected by the age of the months at the time of treatment initiation. The final efficacy evaluation was influenced by the age at the beginning of treatment and the layer of IH.

**Conclusion:**

Oral propranolol combined with local sclerotherapy is a safe and effective method for treating lip IH. After combination therapy, the therapeutic effect of hemangiomas located in the mucosa and submucosa is better than those located in the skin and superficial subcutaneous fascia. Patients who were younger at treatment initiation received less frequencies of topical sclerotherapy and had better therapeutic effect.

## 1. Introduction

Infantile hemangioma (IH) is one of the most common benign tumors in infants, and it has a self-limited course of disease [1]. However, parts of IHs grow rapidly without treatment in the proliferative stage, resulting in ulcers, bleeding, infection, and other complications. Therefore, early active intervention is needed. At present, the treatment methods for hemangioma include oral drugs, topical drugs, topical injection, laser, and surgical resection. In 2008, Leaure-Lebreze et al. noted that propranolol, a nonselective beta blocker, had an effect of inhibiting the growth of IHs [2]. And it has been suggested as a first-line therapy in IH treatment so far [3]. Moreover, direct drug delivery to the tumor is also a common method of treating IH. Lauromacrogol and triamcinolone acetonide are widely used in topical rejection in multiple studies [4–6]. For some patients who are not sensitive to monotherapy, the combination of oral propranolol and topical sclerotherapy can achieve an ideal therapeutic effect to some extent.

Labial region, which has a special histological structure, locates in a rubbed and immersed environment. Therefore, lip hemangioma is more likely to cause ulcer than other parts, resulting in scar, deformities, and even facial damage [7]. Lip hemangioma needs early intervention, but the best therapy is still unclear. To date, there is no clinical study of oral propranolol combined with local sclerotherapy for the treatment of lip hemangioma. Thus, the study is aimed at analyzing the therapeutic effect of combined therapy for the treatment of infantile lip hemangiomas and assessing the main factors that impact the prognosis.

## 2. Materials and Methods

This study was approved by the Institutional Ethics Review Board of Shandong Provincial Hospital (No. 2022-042). We enrolled patients with lip IHs who received the above combination therapy at the Department of Plastic Surgery of Shandong Provincial Hospital from January 2017 to December 2020 for a retrospective analysis. Those who met one of the following criteria were excluded from the study: (i) patients diagnosed with superficial hemangioma according to International Society for the Study of Vascular Anomalies (ISSVA); (ii) patients with platelet crisis, bronchial asthma, sinus bradycardia, severe or acute heart failure, liver and kidney dysfunction, or other drug contraindications; (iii) patients who received other treatments except the combination therapy; (iv) patients over 24 months at treatment initiation; and (v) patients with poor compliance and those who were lost to follow-up.

All patients' parents signed written informed consent. Before treatment, all patients had received ultrasound testing, blood routine examination, electrocardiogram, and other tests to clarify conditions and to eliminate contraindications to treatment. The patients were initially given 1.0 mg/kg ·d propranolol. The dose was increased to 2.0 mg/kg ·d for those with no obvious adverse reactions after 3 days. Topical sclerotherapy was performed in a sterile operating room under general anesthesia. Tessari method [8] was used to prepare the foam with the volume ratio of lauromacrogol to air 1 : 4. The mixture was evenly mixed according to the volume ratio of triamcinolone acetonide and normal saline 1 : 2. The above liquid was injected into the IH at multiple points with the beginning of lauromacrogol foam and then triamcinolone under the guidance of B-ultrasound. The dose was determined by the weight of patients and the size of IH. Generally speaking, the maximum doses of lauromacrogol and triamcinolone were, respectively, 3.5 and 2.0 mg/kg. Patients were asked to return after 4 weeks of topical sclerotherapy and to continue oral propranolol out of hospital. During the review, the patients' clinical symptoms and ultrasound results were used to determine whether to adjust the dosage of propranolol and whether to perform sclerotherapy again. The treatment could be considered to stop when the IH of the patients had basically subsided or the blood flow signal was lower than 20% normally. Before discontinuing treatment, the dose was reduced to 1.0 mg/kg ·d and again 0.5 mg/kg ·d a month later. Patients with no recurrence of IHs after one month of taking 0.5 mg/kg ·d dose can discontinue propranolol. This criterion was not absolute due to the preferences of parents.

Some clinical data should be collected, including sex, age at treatment initiation, locations, subclassification, morphology, thickness, layer, blood flow signal of IH tissues, duration of medication, frequencies of injection, and adverse events. Patients were followed up 6 months after the end of treatment to determine rebound. Photographs of patients at different stages were saved to compare changes in IH size and color. We applied the scale proposed by Achauer et al. [9] to classify the therapeutic effect into 4 grades: I (poor): IH reduction of 0-25%, II (medium): IH reduced by 26-50%, III (good): IH reduced by 51-75%, and IV (excellent): IH reduction > 75%. Furthermore, parents gave marks using the visual analogue scale (VAS) on the scope and color of IH before and after treatment. A positive value indicated an increase in volume, bright color, or filling degree; a negative value indicated a decrease in color, volume, or filling degree; a score of 0 indicated no change in IH.

Statistical analysis was performed through IBM SPSS 25.0. A nonparametric test was used to analyze the relationship between classification variables, grade variables, and therapeutic effect. Spearman correlation analysis was used to statistically analyze the correlation between continuous variables and therapeutic effect. For the convenience of further statistical analysis, sclerotherapy frequency was divided into three grades: 1~3 times, 4~6 times, and 7~9 times, as well as the VAS score was divided into three grades: -2~-4, -5~-7, and -8~-10. In order to exclude the influence of confounding factors, variables with *P* < 0.10 in the univariate analysis were included in multivariate logistic regression analysis to further analyze the factors influencing patient efficacy.

## 3. Results

### 3.1. General Characteristics

Of all 56 patients with infantile lip hemangioma included in this study, 17 (30.3%) were male and 39 (69.6%) were female. The median age at treatment initiation was 4.32 m (IQR: 2.77 m~7.19 m). 14 (25.0%) patients had tumors located in the upper lip, as well as 22 (39.3%) in the lower lip, 9 (16.1%) in the angulus oris, and 11 (19.6%) in the philtrum. A total of 46 (76.8%) patients had single IH, 5 (8.9%) had multiple IH, and 5 (8.9%) had segmental IH. According to the morphology of ISSVA, there were 43 (76.8%) patients with mixed hemangioma and 13 (23.2%) patients with deep hemangioma. The layer and related parameters of hemangiomas were determined by surface ultrasound. According to B-ultrasound localization, IH was located in the skin and superficial subcutaneous fascia layer in 21 (37.5%) patients and in the mucosa and submucosa in 35 (62.5%) patients. The median volume of the tumor before treatment was 1.01 cm^3^ (IQR: 0.61 cm^3^~1.70 cm^3^), and the median blood flow signal was 40% (IQR: 40%~40%) (Tables 1 and 2).

The hemangiomas of 56 cases were controlled to a certain extent after receiving the above combination therapy with no serious complications occurring, such as ulceration. The median duration of oral propranolol was 9.00 m (IQR: 6.25 m~12.00 m). The median frequency of local injection was 3 (IQR: 2.00~4.75).

The Achauer grade ranged from I to IV in 56 patients who received oral propranolol combined with sclerotherapy with lauromacrol and triamcinolone acetonide. Among them, 6 cases (10.7%) were grade I, 12 cases (21.4%) were grade II, 15 cases (26.7%) were grade III, and 23 cases (41.1%) were grade IV.

The subjective evaluation index of the patients' parents, which is namely VAS score, ranged from -2 to -10, of which 9 cases (16.1%) were -2 to -4, 18 cases (32.1%) were -5 to -7, and 29 cases (51.8%) were -8 to -10.16 parents (28.6%) thought that IHs had completely subsided after the combined therapy (i.e., the VAS score was -10).

According to follow-up results after the end of treatment, among all patients included in the study, there was one case of segmental hemangioma with residual after the end of treatment. There were 3 cases of recurrence after drug withdrawal, and the recurrence rate was 5.6%. After laser therapy, all patients with relapsing diseases achieved satisficatory results, and propranolol was not reused. No recurrence or serious complications occurred in the other patients (Tables 3 and 4).

### 3.2. Univariate Analysis

Mann-Whitney *U* analysis showed that there were no statistically significant differences in the duration of the medication, the frequency of sclerotherapy, the Achauer grade, and VAS score among patients of different sex and morphology (*P* > 0.05). There was no statistically significant difference in the duration of taking medicine among patients with different layers of IHs (*P* = 0.296). However, IH in mucosa and submucosa, which received less sclerotherapy (*P* = 0.006), also had a higher Achauer grade (*P* = 0.001) and a lower VAS score (*P* = 0.003) than IH in the skin and superficial subcutaneous fascia.

Kruskal-Wallis H test showed that there were no significant differences in duration and efficacy among patients with IH at various sites of lips (*P* > 0.05). There were statistically significant differences in frequency of sclerotherapy (*P* = 0.017), Achauer grade (*P* = 0.006), and VAS score (*P* = 0.046) among IHs of different classifications. A pairwise post hoc comparison of corrected significance levels using Bonferroni method showed that single IHs had a higher Achauer grade than segmental IHs (*P* = 0.038) and less sclerotherapy than multiple IHs (*P* = 0.049).

Spearman correlation analysis showed that age and volume of IH at treatment initiation were correlated with duration of medication and curative effect. The younger the patients, the shorter the medication (*P* = 0.002), the higher the Achauer grade (*P* = 0.009), and the lower the VAS score (*P* = 0.011). The smaller the IHs, the fewer the frequency of topical sclerotherapy (*P* = 0.024). Furthermore, the smaller IHs also have better curative effects, which means higher Ahauer grades (*P* < 0.001) and lower VAS score (*P* = 0.001) (Table 5).

### 3.3. Multivariate Analysis

Univariate analysis (*P* < 0.10) and clinical correlation were used to identify factors that might affect the treatment process and evaluation of efficacy. According to the above conditions, the classification, the IH layer, the age of the patients, and the volume of IH at the start of treatment were screened as independent variables of the ordered logistic regression analysis. For statistical convenience, the VAS score was divided into three grades, namely, “level 1” (-2~-4), “level 2” (-5~-7), and “level 3” (-8~-10). The frequency of topical sclerotherapy was also divided into three grades: 1~3 times, 4~6 times, and 7~9 times.

The results showed that the age of treatment initiation was the factor affecting the frequency of topical sclerotherapy. For each one month increase in age at the beginning of treatment, the OR value of the increase in injection frequency was 1.240 times (95% CI: 1.025-1.501), *χ*^2^ = 4.907, *P* = 0.027. The age and layer of IHs were the factors that impacted the therapeutic effect. For each one month increase in age at the beginning of treatment, the OR value of Achauer grade decreased by at least one grade was 1.331 times (95% CI: 1.108-1.598), *χ*^2^ = 9.369, *P* = 0.002, and the OR value of the VAS score decreased by at least one grade was 1.353 times (95% CI: 1.105-1.655), *χ*^2^ = 8.586, *P* = 0.003. Meanwhile, compared with IHs located in skin and superficial fascia layer, those located in mucosa and submucosa were at least one grade better in Achauer grade with an OR value of 3.589 times (95% CI: 1.045-12.330), *χ*^2^ = 4.123, *P* = 0.042. The VAS score of IH in the mucosa and submucosa was at least one grade higher with an OR value of 5.789 times (95% CI: 1.493-22.421), *χ*^2^ = 6.454, *P* = 0.011 (Tables 6–8).

## 4. Discussion

The choice of therapy method for IH generally depends on the location, size, depth, stage, and preference of the patients' parents, and lip hemangioma is no exception. However, as a result of lip hemangioma that is easily complicated with ulcers, we need to be more cautious about the dosage and manipulation of the intervention measures for patients. Oral propranolol combined with topical sclerotherapy of lauromacrogol and triamcinolone acetonide was used in this study. Propranolol is undoubtedly the first-line drug in the treatment of IH. The possible mechanism of action is that it acts on the capillary wall and causes hemangioma contraction, blocks the angiogenesis signaling pathway and inhibits cell proliferation, and induces apoptosis of vascular endothelial cells [10–13]. Compared with glucocorticoid, propranolol has a more stable therapeutic effect with fewer adverse reactions and better medication compliance. The combination of oral glucocorticoids is only considered when propranolol is clearly contraindicated at present [14]. However, topical glucocorticoid injection is still widely used due to its small side effects. Lauromacrogol is a hardener that hardens blood vessels by damaging endothelial cells and inducing aseptic inflammation, leading to thrombosis and fibrosis [15]. Common lauromacrogol solution is easily diluted by blood, resulting in shorter contact time between drugs and blood vessel wall, which cannot achieve the desired effect. Therefore, foam hardener is usually prepared by mixing lauromacrogol and air in clinical treatment, thus improving hardening efficiency. The above combination therapy can shorten the duration of the medication, reduce the frequency of sclerotherapy, and inhibit the growth of IH to the greatest extent.

Traditional sclerotherapy injections may cause necrosis of lip tissue and ulceration of lip hemangioma due to overdoses and imprecise injection sites. Therefore, ultrasound-guided injection was adopted in this study. At the same time, we strictly control the dose of drug injection, in line with the treatment principle of less than more. All patients who completed the treatment achieved some degree of improvement of the disease without ulceration and other serious complications, indicating that our drug dosage was safe and reasonable. Figures 1 and 2, respectively, show the therapeutic effects of combined therapy on 2 patients with lip hemangiomas. Furthermore, a patient had residual lesions after treatment, and our center suggested that the patient could be treated with surgery before preschool. The method in which a patient discontinues medication before the end of treatment is also crucial, as tapering may help reduce the rate of rebound compared with outright discontinuation [16]. In our center, we use the method of step-down dose withdrawal. A total of three patients had relapses after finishing treatment and were cured after laser treatment. None of them resumed oral propranolol therapy again. There is no clear standard for the tapering of propranolol, and further studies are expected to provide guidance for the treatment of IH in the future.

The lower lip hemangioma may have higher risk of ulceration than the upper possibly. The reason is that the lower lip receives more friction and dipping during feeding and crying. But among untreated IHs, the prognosis of the upper lip hemangioma may be worse than the lower lip hemangioma [7, 17]. We compared the therapeutic effect of IH in different sites of the lip after receiving the combined therapy. The results showed that the prognosis had no differences in various sites. In addition, Xu et al. [18] suggested that IH across the vermillion boundary had a worse prognosis. In this study, we determined the layer of tumors by ultrasound, which is a more accurate and economical method of localization. The layer was divided into two sorts, in general. The sonographic findings of the skin and subcutaneous superficial fascia layer indicated that IHs were located at white lips to the naked eyes, while mucosa and submucosa on the behalf of red lips. Mucous and submucous hemangiomas were found to receive a better curative effect after treatment. This view is basically consistent with previous studies that have used other treatments. The natural course of IH is known to be somewhat self-limiting. Different treatments lead to similar outcomes. This may indicate that the different prognosis of lip hemangioma is not only affected by the treatment but also related to its self-limiting.

In our study, we found that the age at treatment initiation influenced the duration of the medication, the frequency of sclerotherapy, and the curative effect. Younger patients at treatment initiation mean shorter duration of oral propranolol, the fewer topical sclerotherapy, and better outcomes. That is to say, early intervention of IHs may obtain better therapeutic effect, which is consistent with the research results of our center [19] and some previous studies [20, 21]. Therefore, we recommend early treatment for patients with moderate to high-risk IH. The influence of age on frequency of sclerotherapy did not have statistically significance in the univariate analysis, but the *P* value was less than 0.05 in the multivariate analysis. The reason was possibly that the results of the univariate analysis included the influence and interaction of other variables. Multivariate analysis confirmed the independent effect of age on the frequency of sclerotherapy after eliminating the influence of confounders.

Additionally, in the univariate analysis, the IH classification had an impact on the frequency of sclerotherapy and the curative effect, while this factor was not statistically significant in the multivariate analysis, which may be because the influence of confounders was not excluded in the univariate analysis. Segmental hemangioma is often associated with some syndromes, such as PHACE syndrome [22]. Therefore, the prognosis of segmental hemangioma may be worse than that of single or multiple hemangiomas based on clinical experience. Due to the limited sample size of our study, the specific relationship between segmental hemangioma and the prognosis of patients needed further study.

This study had the following limitations. It is a single-center study, and the sample size of the included study is limited, which may bias the research results. Some data (such as adverse reactions after treatment) were obtained from follow-up visits and recorded by parents themselves due to the study is retrospective, which may be deviated from the actual situation. Finally, IH is a self-limited disease, but our center recommended that children with mixed and deep hemangioma of the lip receive treatment as soon as possible, and we failed to set a blank control group, so that the results of the study have certain limitations.

## 5. Conclusion

In summary, oral propranolol combined with local sclerotherapy of lauromacrogol and triamcinolone acetonide is a safe and effective procedure in the treatments of infantile lip hemangioma. After the above combination therapy, the therapeutic effect of lip hemangiomas located in the mucosa and submucosa is better than those located in the skin and superficial subcutaneous fascia. Patients who were younger at treatment initiation had shorter course of treatment and better outcomes. Future prospective trials involving a larger sample size and a longer follow-up period should be addressed to further clarify our conclusions to provide more accurate treatment to patients with lip hemangioma.

## Figures and Tables

**Figure 1:** Mixed hemangioma of the upper lip before and after therapy.

**Figure 2:** Deep hemangioma of the upper lip before and after therapy.

**Table 1:** Characteristics of the patients (1).

Characteristic	Group	*N* = 56 (%)
Gender	Male	17 (30.3)
	Female	39 (69.6)

Location	Upper lip	14 (25.0)
	Lower lip	22 (39.3)
	Angulus oris	9 (16.1)
	Philtrum	11 (19.6)

Layer	Skin and superficial subcutaneous fascia	21 (37.5)
	Mucosa and submucosa	35 (62.5)

Morphology	Mixed	43 (76.8)
	Deep	13 (23.2)

Classification	Single	46 (82.1)
	Multiple	5 (8.9)
	Segmental	5 (8.9)

**Table 2:** Characteristics of the patients (2).

Characteristics	Minimum	Maximum	Median
Age (m)	1.33	11.80	4.32 (2.77-7.19)
Volume (cm^3^)	0.09	4.60	1.01 (0.61-1.70)
Blood signal (%)	20	50	40 (40-40)

**Table 3:** Evaluation of the curative effect in patients (1).

	Achauer grade				VAS score		
	I (*n* = 6)	II (*n* = 12)	III (*n* = 15)	IV (*n* = 23)	-2~-4 (*n* = 9)	-5~-7 (*n* = 19)	-8~-10 (*n* = 28)
Gender							
Male	1	5	4	7	2	3	12
Female	5	7	11	16	7	15	17
Location							
Upper lip	2	2	4	6	3	4	7
Lower lip	1	6	6	9	2	8	12
Angulus oris	2	2	2	3	2	4	3
Philtrum	1	2	3	5	2	2	7
Layer							
Skin	5	7	5	4	7	9	5
Mucosa	1	5	10	19	2	9	24
Morphology							
Mixed	4	8	12	19	7	12	24
Deep	2	4	3	4	2	6	5
Classification							
Single	3	7	14	22	5	13	28
Multiple	2	2	0	1	2	2	1
Segmental	1	3	1	0	2	3	0

**Table 4:** Evaluation of the curative effect in patients (2).

	Achauer grade (median)				VAS score (median)		
	I	II	III	IV	-2~-4	-5~-7	-8~-10
Age (m)	7.29	8.09	4.53	3.87	8.57	5.69	3.87
Volume (cm^3^)	1.81	1.68	0.75	0.66	1.95	1.05	0.72
Blood signal (%)	40	40	40	40	40	40	40

**Table 5:** *P* value of univariate analysis.

		Oral propranolol duration	Frequency of sclerotherapy	Achauer grade	VAS score
Mann-Whitney *U*-test	Gender	0.245	0.612	0.993	0.310
	Morphology	0.322	0.678	0.256	0.274
	Layer	0.296	0.006	0.001	0.003

Kruskal-Wallis H test	Location	0.833	0.017	0.006	0.046
	Classification	0.979	0.398	0.845	0.285

Spearman correlation analysis	Age	0.002	0.092	0.009	0.011
	Volume	0.097	0.024	0.000	0.001
	Blood signal	0.431	0.946	0.604	0.763

**Table 6:** Multivariate logistic regression analysis of factors that may influence the frequency of sclerotherapy.

	OR	Lower 95% CI	Upper 95% CI	*χ* ^2^	*P*
Age	1.240	1.025	1.501	4.907	0.027
Volume	1.276	0.578	2.824	0.364	0.546
Layer					
Skin	1.092	0.774	11.370	2.518	0.113
Mucosa					
Classification					
Single	0.372	0.034	4.112	0.651	0.420
Multiple	0.196	0.088	38.016	0.152	0.697
Segmental					

**Table 7:** Multivariate logistic regression analysis of factors that may influence Achauer grade.

	OR	Lower 95% CI	Upper 95% CI	*χ* ^2^	*P*
Age	1.331	1.108	1.598	9.369	0.002
Volume	1.640	0.802	3.353	1.837	0.175
Layer					
Skin	3.589	1.045	12.330	4.123	0.042
Mucosa					
Classification					
Single	0.322	0.032	3.241	0.924	0.336
Multiple	1.632	0.090	29.755	0.109	0.741
Segmental					

**Table 8:** Multivariate logistic regression analysis of factors that may influence VAS score.

	OR	Lower 95% CI	Upper 95% CI	*χ* ^2^	*P*
Age	1.353	1.105	1.655	8.586	0.003
Volume	0.505	1.112	4.371	2.881	0.090
Layer					
Skin	5.789	1.493	22.421	6.454	0.011
Mucosa					
Classification					
Single	0.452	0.039	5.233	0.403	0.526
Multiple	0.907	0.042	19.826	0.004	0.951
Segmental					

## Data Availability

The data used to support the findings of this study are available from the corresponding author upon request. Parts of important data will be attached to this submission.
